# Prevalence of sexually transmitted infections and associated risk behaviors in prisoners: A systematic review

This article has been retracted.

**DOI:** 10.1002/hsr2.819

**Published:** 2022-09-15

**Authors:** SeyedAhmad SeyedAlinaghi, Zahra Pashaei, Ensiyeh Rahimi, Solmaz Saeidi, Pegah Mirzapour, Tayebeh Noori, Afsaneh Ghasemzadeh, Arian Afzalian, Mohsen Dashti, Pedram Habibi, Behnam Farhoudi, Narjes Aghaie, Ahmadreza Shamsabadi, Omid Dadras, Esmaeil Mehraeen

**Affiliations:** ^1^ Iranian Research Center for HIV/AIDS, Iranian Institute for Reduction of High‐Risk Behaviors Tehran University of Medical Sciences Tehran Iran; ^2^ Department of Nursing Khalkhal University of Medical Sciences Khalkhal Iran; ^3^ Department of Health Information Technology Zabol University of Medical Sciences Zabol Iran; ^4^ Department of Radiology Tabriz University of Medical Sciences Tabriz Iran; ^5^ School of Medicine Tehran University of Medical Sciences Tehran Iran; ^6^ Social Determinants of Health Research Center, Amiralmomenin Hospital, Tehran Medical Sciences Islamic Azad University Tehran Iran; ^7^ School of Nursing and Midwifery Tehran University of Medical Sciences Tehran Iran; ^8^ Department of Health Information Technology Esfarayen Faculty of Medical Sciences Esfarayen Iran; ^9^ Department of Global Public Health and Primary care University of Bergen Bergen Norway; ^10^ Department of Health Information Technology Khalkhal University of Medical Sciences Khalkhal Iran

**Keywords:** prisoners, risk factors, sexually transmitted disease

## Abstract

**Background and Aims:**

Sexually transmitted infections (STIs) are one of the major health concerns globally. Generally, prisoners are at higher risks for STIs due to risk factors including; drug‐use, high‐risk sexual behaviors, densely populated prisons, and poor living conditions. Therefore, we aimed to conduct a systematic review to evaluate the existing data on STI prevalence, and its associated risk factors among prisoners.

**Methods:**

We conducted a systematic search of the literature using the keywords in Scopus, PubMed, Web of Science, and Google Scholar online databases. We selected all the relevant original studies in English through title/abstract and full‐text screening process.‎

**Results:**

Based on the inclusion and exclusion criteria, we selected and reviewed 32 studies out of 96 identified papers. The most important STI‐associated risk factors among prisoners were drug use, low educational levels, and unsafe sex. The prevalence of STIs was heterogenous in selected studies and was reported as follows; Human Immunodeficiency Virus (HIV) (0%−14.5%), hepatitis B viruses (HBV) (0.04%−27.23%), hepatitis C viruses (HCV) (0.17%−49.7%), Syphilis (0.2%−22.1%), Chlamydia Trachomatis (CT) (1.02%−6.7%), Gonorrhea (0.6%−7.8%), and herpes simplex virus‐2 (HSV‐2) 22.4%.

**Conclusion:**

This systematic review indicates that the prevalence of STIs (HIV, HBV, HCV, Syphilis, Chlamydia Trachomatis, Gonorrhea, and HSV‐2) among prisoners appears to be higher than the general population, with drug abuse, low educational levels, and unsafe sex as major risk factors.

## 1 INTRODUCTION

Sexually transmitted infections (STIs) place an extensive burden on sexual and reproductive health worldwide. Although, more than 30 pathogens are recognized to be sexually transmitted, eight of these have been noticeably associated with a significant rate of morbidity, and mortality.^1^ Three bacterial STIs, namely Chlamydia trachomatis (CT) (chlamydiasis), Neisseria gonorrhoeae (gonorrhea), and Treponema pallidum (syphilis), and one parasitic STI, Trichomonas vaginalis (trichomoniasis), are currently curable, while five viral STIs, Human Immunodeficiency Virus (HIV), human papillomavirus, herpes simplex virus (HSV), and hepatitis B and C viruses (HBV and HCV), can be chronic or lifelong, although medications can modify disease course or symptoms.^1^

According to the latest report from World Prison Population List (13th edition) by Helen Fair, and Roy Walmsley, by the end of 2021, there were an estimated 10.7 million people incarcerated across the world. Since 2000, the estimated world prisoner population has been increased by about 24.3%.^2^ Accumulation of negative health risks and precarious living conditions in prisons such as sedentary lifestyle, poor diets, inadequate hygiene habits, and drug use contribute to the transmission of infectious diseases among prisoners.^3^ High‐risk transmission behaviors like continuing drug injection and syringe‐sharing, unsafe sexual behavior, tattooing, and piercing in a prison setting can lead to quick and severe disease transmission and progression.^4^, ^5^

Incarcerated people make up a key population group of societies that are at high risk of being infected with STIs and blood‐borne infections, especially Persons Who Inject Drugs (PWID) that comprise of approximately 3%−50% of prisoners.^6^ Viral STIs such as HIV/Acquired Immunodeficency Syndrome (AIDS), HBV, HCV, and bacterial STIs such as Chlamydia trachomatis, Neisseria gonorrhoeae, and Treponema pallidum (syphilis) share the same transmission root but have different burdens and costs.^7^, ^8^ Viral STIs have asymptomatic initiation and may remain undiagnosed for many years.^9^ Bacterial infections may be also asymptomatic and they are curable with short courses of antibiotics.^10^, ^11^

Since almost all prisoners are eventually released, the potential for continuous transmission of STIs in the free society has significant implications for public health. Mathematical models suggests that half of all HIV new cases among PWID in Eastern Europe and Central Asia could be attributed to a history of incarceration.^12^ Therefore, identification and early treatment of infected inmates is fundamental not only to limit the disease burden and costs within the prison but also to reduce the risk of STI transmission to the general population upon the release from prisons. Besides, prisoners are not a static population and often move back and forth to the outside world and could circulate the infection.^13^ This indicates a considerable gap exist in understanding the scale of the problem and in prevention efforts. In fact, prisons provide various conditions for both the spread^4^ and prevention of STIs.^6^

This study provides two important advantages: first, to understand the scale of this public health problem, and second, help health care providers and policy makers develop new effective strategies for solving this problem renewed focus on the target key population, reliable incidence, and prevalence, and specifying risk factors are needed. To accurately, understand the true scale of this public health problem, and to develop new effective strategies for control and prevention, we need; prison‐related risk factor identification, and more reliable prisons STI incidence and prevalence rates compared to the general population. Therefore, we aimed to systematically review the prevalence of STIs and associated specific risk factors among the incarcerated populations worldwide reviewing the relevant articles that have been published until November 2021.

## 2 METHODS

This study is a systematic review of current literature concerning the prevalence and related risk factors of STIs in prisoners. We searched and retrieved the most relevant literature using the keywords in the online databases of Scopus, PubMed, Web of Science, and Google Scholar. All relevant studies in English from January 2015 to November 2021 were included. This review adhered to the Preferred Reporting Items for Systematic Reviews and Meta‐Analyses (PRISMA) statement.

### 2.1 Search strategy

A comprehensive search was performed to retrieve articles published in the aforementioned databases. We used multiple combinations of keywords to construct the search strings, some examples are as follows:

(A) “Sexually Transmitted Infections” OR “Sexually Communicable Infections” OR “STIs” OR “Sexually correlates” OR “transmitted disease” [Title/abstract/keywords].

(B) Prisoners OR prison OR incarceration OR imprisoned OR inmates [Title/abstract/keywords].

(C) [A] and [B].

### 2.2 Selection study and data screening

The EndNote X9 software was used to organize the retrieved articles. Search results from databases were combined in a single EndNote library and duplicate articles were removed. Two authors independently screened the retrieved records in different two steps. First, the title and abstract of the articles were screened based on eligibility criteria and relevancy of the content, and the ineligible records were removed. The full texts of the remaining articles were reviewed based on inclusion and exclusion criteria and the eligible studies were recognized. English language, original articles, and the relevance of the articles to the purpose of the study were selected as the inclusion criteria.

We also excluded the publications that met at least one of the following criteria:

1. Unavailability of full texts.
2. Nonoriginal literature includes reviews, conference abstracts, abstract papers, editorials, and meta‐analyses.
3. Ongoing clinical trials without yet published results.
4. Duplications and/or concern about the reliability of results.

### 2.3 Data extraction

Three authors extracted the necessary information for the included studies such as first author's name, type of study, country of study, gender, age, race, marital state, education level, drug use, unsafe sexual history, syndromic diagnosis, etiologic diagnosis, and other findings and enter this data into a spreadsheet. This sheet was designed by the corresponding author. To avoid any probable duplications and/or crossovers, the selected studies were also reviewed by the first author.

### 2.4 Quality assessment

We used the PRISMA statement to report the results of the present review. The quality of the studies was assessed by two independent and expert authors. Any discrepancy or disagreement was addressed by a third independent author.

## 3 RESULTS

In this study, 96 documents were identified using a systematic search strategy. After an initial review of the retrieved articles, 20 duplicates were removed and the titles and abstracts of the remaining records were assessed. After applying the selection criteria, 44 articles were deleted in the two‐phase screening process and 32 articles met the inclusion criteria and were included in the final review (Figure 1).

**Figure 1:** Search results from different databases

Most of studies were cross‐sectional (*n* = 23), following with cohort (*n* = 8), and randomized control trial (*n* = 1). These studies were conducted in 17 countries. Eight studies were from Brazil, five studies from USA, two studies from each of Ethiopia, and Iran, and one from each of the following: Myanmar, France, Benin, Kyrgyzstan, Indonesia, Mexico, Belgium, Spain, Swiss, South Africa, Germany, Nigeria, and Italy. Also, a study was conducted in several countries from European Union, European Economic Area, and the United Kingdom.

Reviewing the included records, it appeared that the most important risk factors in prison are the high‐risk behaviors that harm the STIs prevention programs apart from having a history of STIs. Single inmates were more likely to suffer from STIs than married inmates. Most inmates were illiterate or had a low education level. In almost all studies, having a history of substance abuse was statistically significant among inmates suffering from STIs. This review documented HIV, HBV, HCV, and syphilis as the most frequent STIs among prisoners (Table 1).

**Table 1:** Prevalence of STIs and associated factors in prisoners

ID	The first author	Type of study	Country	Factors related to the prevalence of sexually transmitted infections in prisoners								
				Gender (%)	Age (mean)	Race/ethnicity	Marital state	Educational level (%)	Drug use (%)	Unsafe sexual history (%)	Syndromic diagnosis	Etiology (%)
1	Rachel et al.^14^	Cross‐sectional	Indonesia	Female: (100)	33.4 ± 9.9	Indonesian	Married: (56) Divorced: (28.5) Single: (15.5)	No education: (5.1) Low education: (36) High education: (58.9)	Alcohol: (26.2) Drug: (6.8)	55.6	Serosurvey	HIV: (3.7) Syphilis: (7.0) HBV: (3.3) HCV: (2.3)
2	Azbel et al.^15^	Cross‐sectional	Kyrgyzstan	Female: (13) Male; (87)	Female: 40.6 ± 9.1 Male: 36.8 ± 8.9	Kyrgyz Russia Uzbek	N/A	Completed high school: (77)	Opioid use Ever injected drug Sedatives use	N/A	HIV: ELISA test by Western blot testing HBV: Serosurvey HCV: Serosurvey Syphilis: RPR titer ≥ 1:16	HIV: 10.3 HBV: 6.2 HCV: 49.7 Syphilis: 19.2
3	Batista et al.^16^	Cross‐Sectional	Brazil	Female: (100)	29.8 ± 8.2	Mixed race: (54) White: (32.7) Black: (11.5) Yellow: (1.8)	Single: (63.7) Married: (25.7) Divorced: (8.8) Widowed: (1.8)	None: (7.1) 1−3 years: (24.8) 4−7: (37.2) 8−11: (18.6) 12 or more: (12.4)	Injectable drugs: (50.4) Alcoholic beverages: (64.6)	Use of condom/casual (34.4) Use of condom/fixed partner (8.1)	The combination of recombinant *Treponema Pallidum* antigens bound to a membrane (solid phase) and protein A conjugate with colloidal gold particles Quick Test Form proposed by the Ministry of Health on risk situations for STI	Syphilis: (22.1)
4	Bautista‐Arredondo et al.^17^	Cross‐Sectional	Mexico	Female: (10.2) Male: (89.8)	Female: 34.9 ± 10.2 Male 33.1 ± 9.3	Mexican	N/A	Less than 10 years of formal education (male: 71.4, female: 62.2) University level: (male: 7.2, female: 16.7)	Illicit substances (male: 69.9, female: 59.1) Injected drugs (male: 5, female: 3.7) Injecting nonprescribed vitamins (Male: 48.4, female: 55.1)	Condom use: (male: 20.5 female: 18.3)	Blood samples HIV: 1 and 2 antibodies‐p24 antigen by Abbott Architect Ag/Ab Combo Hepatitis B: antibody (HBcAb) by Abbott Architect Anti‐HBC II‐ Hepatitis B surface antigen (HBsAg) Hepatitis C: Antibodies by Abbott Architect Anti‐HCV Syphilis: antibody (Anti‐TP) by Abbott Architect Syphilis TP‐Venereal Disease Research Laboratory (VDRL)	Female HIV: (0.8) HCV: (2.6) Hepatitis B: (3.3) Syphilis: (3.3) Male HIV: (0.7) HCV: (3.3) Hepatitis B: (2.9) Syphilis: (1.8)
5	Benedetti et al.^18^	Cross‐sectional	Brazil	Female: (100)	36.5 ± 9.5	Brazilian	Married: (28.6), Single: (50) Steady relationship: (7.75) Widowed: (2.4) No information available: (11.3)	Illiterate: (11.9)	N/A	Not used condoms: 59 (39.6)	HIV: HIV‐1/2 specific antibodies Syphilis: IgG, IgM and IgA antibodies against *Treponema pallidum* hepatitis B: HBs antigen	HIV: (4.7) Syphilis: (15.5)
6	Busi. et al.^19^	Cross‐sectional	Ethiopia	Female: (20) Male: (80)		Ethiopian	Not married: (52.6) Married: (36.4)	Education above 12th grade: (30.3) Secondary school education: (27.55)	Alcohol and cigarettes: (21), Substances: (20.9)	N/A	Burning sensation during urination Sore penis Sore vagina Abnormal genital discharge Pain during or after sexual intercourse while vaginal discharge Bleeding or blood spotting from the vagina Thick, cloudy, or strong vaginal Odor discharge from the vagina Vaginal itching or irritation Abnormal menstrual bleeding	HIV: (14.5)
7	Busschots et al.^20^	Cohort	Belgium	Male: (93) Female: (7)	Birth date: 1981 ± 1974–1990	Belgian	N/A	N/A	Used heroin in last 6 months (10.6) Used drugs in last 6 months: (68.7)	N/A	HIV: HIV Ab/Ag HCV: OraQuick Ab HBs: HBs Rapid device Ag BBV: questionnaire	HIV: (0.2) HCV: (5) HBs: (0.8)
8	Carnicer‐Pont et al.^21^	Cross‐sectional	Spain	Male: (93.4) Female: (6.6)	Male: (40) Female: (39.5)	Spanish	N/A	Secondary level: (43) University level: (9)	Drug consumption: (75)	N/A	Serostatus	HIV: (7.9) HCV: (13) HBS: (27.8) STI: (5.3)
9	Chacowry Pala et al.^22^	Cross‐sectional	Swiss	Male: (100)	29.8 ± 9.0	Central and Eastern Europe, Sub‐Saharan Africa, North Africa, Latin America, Western Europe, Asia	N/A	Secondary school not completed: (27.9) Secondary school completed: (72.1)	N/A	N/A	HIV: Ag/Ab Combo, Architect, Abbott HCV: anti‐HCV, Architect, Abbott HSV: HSV‐2 IgG enzyme‐linked Immunosorbent assay (ELISA) (Immunowell, HSV type 2, IgG test, GenBio	HIV: (0.4) Syphilis: (1.2) HSV‐2: (22.4) HCV: (6.2)
10	Defante Ferreto et al.^23^	Cross‐sectional	Brazil	Male and female	32.58 ± 10.18	White, Asian, Brown, Black, Indigenous	Single: (53.3) With someone: (46.67)	Incomplete primary education: (95.5) Complete primary education: (4.415)	Injecting drug: (13) Alcohol: (26)	N/A	HIV: Geenius^TM^ HIV 1/2 confirmatory assay and Western Blot HCV: Anti‐HCV high throughput chemiluminescent microparticle immunoassay	HIV: (2) HCV: (3.1) STI: (15.2)
11	do Nascimento et al.^24^	Cohort	Brazil	Male and female	18 and above	N/A	Single: (45.3), Married: (41.2), Divorced: (7.1), Widow: (2)	Illiterate: (2.56) Incomplete elementary school: (47.24), Complete elementary school: (17.14), Incomplete high school and/or technical education: (16.60), Complete high school and/or technical education: (9.32), Incomplete university: (1.49), University graduate: (1.08)	N/A	N/A	Tuberculosis: cough for ≥2 weeks, regardless of other clinical manifestations) chest X‐ray examination HIV: RT1 and RT2‐enzyme immunoassay, western blot, immunoblot (IB), or inline immunoassays HBV, HCV: HBsAg total anti‐HBc IgM and IgG classes, anti‐HBs, HBeAg and anti‐HBe—HBV‐DNA viral load (DNA of HBV). Syphilis: anti‐*Treponema pallidum* antibodies	HIV: (0.68) TB: (0.66) Syphilis: (0.2) HCV: (0.17) HBV: (0.04)
12	El Maerrawi et al.^25^	Cross‐sectional	Brazil	Male: (100)	29.8	Brown, Black, White, Yellow and Indian	N/A	Illiterate: (1.5) schooled for fewer than 8 years: (73) schooled for more than 8 years: (25.5)	Among illicit drug users; Cocaine: (87.6) Heroin: (6.2) Other drugs and opiates: (6.2)	N/A	HIV: ELISA kits‐ immunoblot kits HCV: ELISA kits‐ immunoblot kits HBs‐Ag, HBeAg, anti‐HBeAg, HBV: anti‐HBc, anti‐HBcIgM and anti‐HBs Syphilis: HBs‐Ag, HBeAg, anti‐HBeAg, HBV: anti‐HBc, anti‐HBcIgM and anti‐HBs	HIV: (1.8) HBV: (21) HCV: (5.3) Syphilis: (5.3)
13	Felisberto et al.^3^	Cross‐sectional	Brazil	Male: (100)	18−55	N/A	N/A	Illiterate: (2.8) Incomplete fundamental school: (57.2) Complete fundamental school: (15.9) Incomplete high school: (10.3) Complete high school: (13.9)	Injected drug use: (4.8%)	N/A	HIV: fast immunoblotting technique	HIV: (2.1)
14	Getachew et al.^26^	Cross‐sectional	Ethiopia	Male: (79) Females: (21)	18–29	Gamo, Gofa, Oyda, Gidicho, Zeyse	Unmarried: (59.3), Married: (30), Widowed: (6.7), Divorced: (4)	Grade 1–4: (24.8), Grade 5–8: (49.4), Grade 9–10: (11.9), Grade 11–12: (13.9).	Alcohol use: (20.7)	Without condom: (4)	Self‐Reported Syndromes of STIs: Urethral discharge in men Genital ulcer Vaginal discharge Lower abdominal pain in women Inguinal bubo (swelling in the groin region), an Scrotal swelling	Abdominal pain: (25.5) Scrotal swelling: (57.1) Inguinal bubo: (8.6) Urethral discharge: (85.7) Vaginal discharge: (14.3) Genital ulcers (40)
15	Hessou et al.^27^	Cross‐sectional	Benin	Male: (83.5) Female: (16.5)	14−80	Benin, Ghan, Togo, Niger	Unmarried (no partner: (25.25), Unmarried (one or multiple partners): (14.5), Married: (54.3), Divorced/Widow: (4.2)	None: (30.9) Primary: (27.9) Secondary and higher: (41.2)	Alcohol: (56.2) Injectable drugs: (6.3)	N/A	Blood samples and behavioral questionaire	HIV: (1.4)
16	Izquierdo^28^	Cohort	France	Male: (90) Female: (10)	18−80 (31)	Westen European, Middle East, North Africa, and Greater Arabia, Central and South America, Sub‐Saharan Africa, Eastern Europe, Asia	N/A	N/A	N/A	N/A	For anti‐HEV: (IgG) and M (IgM) using the Wantai HEV‐IgG ELISA and HEV‐IgM ELISA kit. for HIV, HAV, and HCV (HBsAg), (anti‐HBs) and (anti‐HBc) using the HIV combi PT, Anti‐HAV, Anti‐HCV II, HBsAg II, Elecsys Anti‐HBs II, and Elecsys Anti‐HBc II electrochemiluminescence immunoassays kits.	HEV: (8.2) HIV: (1.3) HAV: (62.7) HBV: (1.9) HCV: (2.9)
17	Khademi et al.^29^	Cross‐sectional	Iran	Male: (100)	35.52 ± 8.12(19−64)	Iranian	HBSAG+ Single: (38.5), Married: (30.8), Divorce: (30.8) HCVAB+ Single: (51), Married: (33), Divorce: (16.1) HIVAB+ Single: (59.4), Married: (12.5), Divorce: (28.1)	N/A	Current cigarette smokers: (85) History of hookah smoking: (35.4) Substance use: (93) Alcohol drinking: (78)	N/A	The (ELISA) was performed as A confirmatory test for cases with positive results in the rapid test. Seropositive samples for hepatitis B antigens and hepatitis C antibodies were considered positive Hepatitis B and hepatitis C patients, respectively. Individuals with one positive rapid test and two positive ELISA tests were considered positive for AIDS.	The seroprevalences: HBV: (1.25) HCV: (22.2) HIV: (3.09)
18	Khan et al.^30^	Cohort	USA	male	34.4 (SD9.6)	African American	Married: (19) Lived with partners: (61) Helped their spouse pay for Demands: (87) Received help paying for needs from partners: (83)	N/A	Illegal drug use: (55) Noninjection drug use: (54) Ever injected drugs: (4.8)	N/A	Blood sample	All people were HIV‐negative
19	Khan et al.^31^	Cohort	USA	male	36.9 ± 9.6	African American	Married: (23.8) Not‐married: (76.2)	Completed high school: (67.4) Not complete high school; (32.6)	Marijuana use: (60.2) Crack/cocaine use: (48.2)	N/A	Blood sample	N/A
20	Krieger et al.^32^	Cohort	USA	Male	39.1 ± 10.6	Black, White, Hispanic	Ever married: 24.8	N/A	Opioid use: 42.6 Meth: 14.7	N/A	For GC/CT (urine sample, nucleic acid amplification test [NAAT]) Syphilis: RPR HBV: HBsAg and HIV VL. patient with urogenital symptoms (dysuria, discharge, lesions) at time of STI diagnosis, it was recorded as asymptomatic infection	Gonorrhea: (3) Chlamydia: (4) Syphilis: (21) HBsAg: (5)
21	Lederman et al.^33^	Cross‐sectional	USA	Male: 83.1 Female: 16.5 Gender nonconfirming: 0.4	18−78 (28)	N/A	N/A	N/A	Substance use: 16.7 No substance use: 83.3	N/A	Tests conducted were HIV 1/2 fourth‐generation assay (antigen and antibody), hepatitis B surface antigen test, *Treponema pallidum antibodies*: rapid plasma regain *Neisseria gonorrhea* and *Chlamydia trachomatis*:, nucleic acid testing (urine)	STI: (8.5), Positive for >1 STI: (0.5) Chlamydia: (6.7) Syphilis: (0.8) Gonorrhea: (0.6) Hepatitis B: (0.2) HIV: (0.2).
22	Martins et al.^34^	Cross‐sectional	Brazil	Female	Older than 18 years	Caucasian: 41.5 mixed race: 42.1	Partner/12 months 1 partner: (59.2) >1 partner: (40.8)	Incomplete: primary: (31.3) Primary education: (10.6) Incomplete high school: (31.9) High school: (17.2) Some College: (6.3) College; (2.6)	Use alcohol: (60.6) Drugs: (20.4)	Condoms use: Never: (59.6) Sometimes: (41.1) Always: (2.0) Sex for money: (22.7) Sexual violence: (31.9)	STD diagnosed by a physician currently or in the past.	STD: (41.2)
23	Moradi et al.^35^	Cross‐sectional	Iran	Male: (97.3) Female: (2.4)	36.29 ± 10.05	Iranian	Married : (45.35)	nonacademic education: (91.88)	Use drug: (72) Injecting drug use: (15) Shared needles: (37) Tattooing: (48) Extramarital sex: (58)	N/A	HBV and HCV	HCV antibodies: (8.21) HBV antibodies: (3.06)
24	Muller et al.^36^	Cross‐sectional	Germany	N/A	N/A	N/A	N/A	N/A	N/A	N/A	Substances unique to or typically used for the treatment of each disease were defined as a marker substances with defined daily doses (DDD)	The HIV adTP: (0.06 −0.94) HCV adTP: (0.03 −0.59) OST adTP: (0.7−0.9) The overall adTP for the respective treatment: HIV: (0.39) HCV: (0.12) OST: (2.18)
25	Nakitanda et al.^37^	Cohort	European Union, European Economic Area, and the United Kingdom	N/A	N/A	Bulgaria Croatia Finland France Hungary Ireland Italy Luxembourg Portugal Romania Slovakia Spain UK	N/A	N/A	N/A	N/A	serosurvey	Hepatitis B surface antigen sero‐prevalence: (0−25.2)
26	Nom et al.^38^	Cohort	Myanmar	Male: (90.2) Female: (9.8)	32	N/A	N/A	Literate: (85.5)	Inject drugs: (68)	N/A	N/A	HIV+: (5)
27	Okafor et al.^39^	Cross‐ sectional	Nigeria	Male: (90.8) Female: (9.2)	33	N/A	Married: (39.4) Single: (56.3) Divorced: (1.4) Separated; (1.4) Widowed: (1.4)	Primary: (15.5) Secondary: (53.5) Tertiary: (26.8) Nonformal: (4.2)	Injection drug use: (19)	N/A	With blood for diagnosis antibodies to hepatitis C virus	HCV: (29.6)
28	Puga et al.^40^	Cross‐sectional	Brazil	Male: (100)	29	White: (26) Multiracial: (53) Black: (18.7) Asian: (1.4)	With a steady partner: (39.2) Without a steady partner: (57.6)	4 and less than 4 years: (68.5) More than 5 years: (21.1)	N/A	N/A	N/A	HCV: (4.7) HCV RNA: (84.6) HIV: (19) hepatitis B: (9.3) syphilis: (10)
29	Sanarico et al.^41^	cross‐sectional	Italy	Male: (66) Female: (3)	43	N/A	N/A	N/A	Drug abuse (injective and/or noninjective): 78.3%	Heterosexual: (29) homosexual: (2.9)	N/A	HIV‐positive: (92.8) HBV: (81.2) HCV: (81.2) HCV: (42)
30	Silva et al.^42^	cross‐sectional	Brazil	Male (92.8)	30.9	N/A	Single, separated or widowed: (58.8)	Primary education: (63.0)	Alcohol: (81.8) drugs: (72.7)	N/A	The rapid test for Hepatitis B	HBSAG + (0.5)
31	Stephens et al.^43^	Cohort	South African	Male	28.7	Black: (96.7) Caucasian: (0.8) Indian: (0.8) Mixed: (1.70	Single: (76.3) Married: (23.7)	Grade 7: (24.8) Grade 8: (12.4) Grade 9: (34.7) Grade 12: (19) Technical/college: (1.7) No education: (7.4)	N/A	N/A	N/A	N/A
32	Williams et al.^44^	Randomized controlled trial	USA	Male	45	Control: Black, non‐Hispanic, Hispanic, White, non‐Hispanic Intervention: Black, non‐Hispanic, Hispanic, White, non‐Hispanic	Control: Single (62.4) Married (12) Divorced (20.8) Intervention: Single (63.1) Married (16.2) Divorced (16.9)	Control 12 and less 12 years: (20) High school diploma: (60) Technical school/associate's degree: 15.2 Bachelor's degree or higher: 2.4 Other: 1.6 Intervention 12 and less 12 years: 29.2 GED/high school diploma: 55.4 Technical school/associate's degree: 10 Bachelor's degree or higher: 4.9 Other: 1.2	N/A	N/A	N/A	All person were HIV‐negative. Gonorrhea: (7.8) Chlamydia: (4.6) Syphilis: (4.7) Genital warts: (0.8) Herpes: (1.5)

Abbreviations: CT, Chlamydia Trachomatis; GC: Neisseria gonorrhea; HBc, Hepatitis B Virus core; HBV, hepatitis B viruses; HCV, hepatitis C viruses; HSV, herpes simplex virus; IgG, immunoglobulin G; RPR, Rapid Plasma Reagin; STD, sexually transmitted disease; TB, Tuberculosis.

## 4 DISCUSSION

In this systematic review, we investigated the STI prevalence and associated risk factors in incarcerated populations worldwide. In almost all included studies, at least one type of STI was reported among prisoners. The STI prevalence rates in selected studies was heterogenous, and reported as follows; HIV (0%−14.5%), HBV (0.04%−27.23%), HCV (0.17%−49.7%), Syphilis (0.2%−22.1%), Chlamydia Trachomatis (1.02%−6.7%), Gonorrhea (0.6%−7.8%), and HSV‐2 22.4%.

On the other hand, according to the latest reports by Joint United Nations Program on HIV/AIDS (UNAIDS), the global prevalence rate for HIV in general population was estimated at 0.7% in 2021, with infected case rising remarkably from 30.8 million to 38.4 million from 2010 to 2021.^45^ In addition, in 2019 it was measured that hepatitis B have infected more than 316 million people, and its all‐age prevalence rate was estimated to be 4.1%.^46^ Also, the global prevalence of hepatitis C has been estimated to be at approximately ∼3% of the world's population, infecting 150–200 million people.^47^, ^48^ And finally, World Health Organization have reported the global prevalence of curable STIs among adults (15–49 years old) in 2020 as follows; Chlamydia (4%), Gonorrhoea (∼1%), Trichomoniasis (∼5%), and Syphilis (∼1%).^49^ Thus, in comparison to the mentioned global prevalence rates, it seems obvious that STIs were more common among incarcerates compared to the general population.

To find plausible explanations for this discrepancy in this special sub group compared to the general population, some studies had searched for risk factors and stated illicit drugs abuse (specifically IV injections), alcohol abuse, unsafe sex, single marital status, multiple sex‐partners, and low educational levels as possible associated risk factors of higher STI prevalence rates among prisoners. The condition of sexual activity in prisons is largely unknown and suggested to be significantly under‐reported, and screening is not routinely performed among prisoners.

### 4.1 Educational level

In our analysis of 32 publications, 23 papers evaluate the prisoners' educational levels.^3^, ^14^, ^15^, ^16^, ^17^, ^18^, ^19^, ^21^, ^22^, ^23^, ^24^, ^25^, ^26^, ^27^, ^30^, ^34^, ^35^, ^39^, ^40^, ^42^, ^43^, ^44^, ^50^ Most papers had reported that the majority of their participants in the survey/research had low levels of education in comparison to the general population, and mostly only had completed some years of primary/elementary education. Prisoners with no history of institutional education (illiterate) were mentioned by nine articles, and the rate of complete illiteracy among participants ranged from 1.5% to 30.9%.^3^, ^14^, ^16^, ^18^, ^24^, ^25^, ^27^, ^39^, ^43^ In addition, eight articles reported that their sample participants had only completed high school education, with a percentage ranging from 9.32% to 60%.^3^, ^15^, ^16^, ^19^, ^24^, ^26^, ^31^, ^34^, ^44^ Finally, only eight studies reported higher educational levels among their participants, and reported university/college education from a low of 2.5% to a peak of 16.7%.^14^, ^16^, ^17^, ^21^, ^24^, ^34^, ^43^, ^44^ One study reported that, more than 58% had of their participants' high education.^14^ In one included study, 95.5% of incarcerated people had incomplete primary education.^22^ One similar article, noted that people with history of incarceration, are two‐times higher risk to have no high school degree, and approximately 50% of former prisoners, hold only a high school diploma.^51^ Another similar study conducted in Brazil, reported that less than 13% of the prisoners have education accessibility, and among approximately 700,000 inmates, 8% were illiterate, 70% did not finish primary school, and 92% did not finish high school, and less than 1% of inmates had the chance to enter colleges.^52^ Another article indicated that, in the United States approximately, 41% of inmates in 1997 and 31% of probationers did not finish high school while, in comparison, a significantly lower level of 18% of the general population had not finished the 12th grade.^53^ Another study in the United States showed that 30% of prisoners had achieved less than a high school degree which was twice the general percentage for United States households (14%).^54^

All the aforementioned information would be indicative of association of poor educational levels with poor general knowledge in regard to STIs diagnosis, prevention, treatment and routes of transmission. One study in Saudi Arabia, indicated that 83% of prisoners were not aware of STIs, and 57.4% were not screend for STIs.^55^ Other similar studies have also reported poor knowledge of STIs among inmates compared to general population globally; in one study in Italy only 12% of the prisoners had correct knowledge about STIs, in one study Nigeria, 39.5%, 48.7%, and 11.8% of the inmate participants had good, fair and poor knowledge of HIV/AIDS respectively.^56^, ^57^, ^58^ All these information, indicates that poor educatonal levels, and the subsequent poor knowledge of STIs can be a hazardous risk factor for developing STI in prisons globally, and educational, and informative programs can be a good way to address this issue.

### 4.2 Alcohol and drug use

In total, 23 studies, reported alcohol or illicit drugs abuse in their study population.^3^, ^14^, ^15^, ^16^, ^17^, ^19^, ^20^, ^21^, ^23^, ^25^, ^26^, ^27^, ^29^, ^30^, ^31^, ^32^, ^33^, ^34^, ^35^, ^39^, ^41^, ^42^, ^50^ In regard to alcohol, nine studies reported different rates of alcohol consumption among their incarcerated participants with rates ranging from 20.7% to 81.8%.^14^, ^16^, ^19^, ^23^, ^26^, ^27^, ^29^, ^34^, ^42^ In addition, 22 studies indicated illicit drug abuse in their study population ranging from 6.3% to 78.3%,^3^, ^14^, ^15^, ^16^, ^17^, ^19^, ^20^, ^21^, ^23^, ^25^, ^27^, ^29^, ^30^, ^31^, ^32^, ^33^, ^34^, ^35^, ^39^, ^41^, ^42^, ^50^ and six studies specified IV drug abuse rates in their population that was between 6.3% and 68%. In one study conducted in Taiwan, 62.8% (570/908) of inmates were IV drug abusers, and among them HIV had a high prevalence of 21.6%.^57^ In one systematic review of 23 articles, shared contaminated needles for IV drug use was reported as one of the principal hepatitis transmission routes among prisoners.^59^ In another study carried out in Nigeria, 29.6% of inmates who used injection drugs were HCV positive.^39^ Similarly, one large study among 1336 inmates in Ghana, indicated intravenous drug use, history of sharing syringes and drug paraphernalia, as independent determinants for HIV, HBV, and syphilis.^60^ Another large study among inmates in Italy, found that 30.4% of sample population were intravenous drug users, and it was strongly associated with HCV, and HIV infection.^61^

These clearly show that history of drug uses‐specifically IV drug injection‐can be a strong predisposing factor to STI infection.

### 4.3 Unsafe sexual history

In this review, seven studies discussed findings on condom use, or unsafe sexual activities.^14^, ^16^, ^17^, ^18^, ^26^, ^34^, ^41^ Four studies reported their findings on condom use, and condom usage was reported between 18.3% and 60.4%. One of our included articles, reported that the use of condom among inmates with casual partner was 34.4%, and condom use among inmate with a fixed partner was as low as 8.1%.^16^ Another study in Brazil among female inmates reported, 59.6% have never used condoms, 22.7% of incarcerates had sex for money, and 31.9% reported sexual violence.^34^ One large study in Ghana, stated that history of homosexuality, paid sexual activity were independent determinants for developing HIV, HBV and syphilis infection.^60^ In one study in India, among 240 inmates, 76.6% had a history of sex with their wives or casual sex partners, and sex workers.^62^ On study in Nigeria among 300 prisoners, indicated that intraprison anal sex, having multiple sex partners as risk factors for HIV and HBV infection. They also mentioned STIs' transmission routes ignorance as a risk factor for HBV and HCV infection.^63^ One large study in Iran among a total of 5508 prisoners, reported 55% rate of had unsafe sex in their lifetime, of whom 53.4% had never used condoms during mentioned unsafe sex.^64^ Another large study among 5530 inmates in Iran, reported that only 24.7% of participants had used condom at last vaginal/anal sex in prison.^65^ Thus, unsafe sexual behavior in prisons due to poor access to preventive methods, and poor general knowledge of STIs is an important risk factor for developing STIs.

### 4.4 Diagnostic methods

In this systematic review, we investigated 32 studies conducted among prisoners in different regions of the world. Among these studies, three cross‐sectional studies and one RCT only used clinical questionnaires and sign and symptoms self‐reports to assess the prevalence of STDs in their inmate population.^19^, ^21^, ^26^, ^44^ While the remaining 28 studies utilized at least one laboratory diagnostic test or more to confirm and evaluate the STIs among their participants. Among these studies, four mentioned only “blood sample” in their published full‐text article and did not note the specific diagnostic test used.^26^, ^27^, ^30^, ^31^, ^44^ The remaining 24 studies' diagnostic methods are reported below.

### 4.5 HIV

According to Centers for Disease Control and Prevention (CDC), there are five major types of tests available for HIV diagnosis including; Nucleic acid laboratory test, antigen/antibody (Ag/Ab) laboratory test, Ag/Ab rapid test, Ab laboratory test, and Ab rapid test. CDC also signifies that Ag/Ab enzyme‐linked Immunosorbent assay (ELISA) test is the most sensitive and specific test, currently available.^66^

Fifteen studies assessed HIV prevalence among prisoners as follows; the most common laboratory diagnostic methods for HIV detection were HIV 1/2 specific antibodies and HIV Combo Ag/Ab ELISA tests.^14^, ^15^, ^16^, ^17^, ^18^, ^19^, ^20^, ^22^, ^23^, ^25^, ^28^, ^29^, ^33^, ^40^, ^50^ The next common tests were the rapid HIV test^14^, ^29^, ^50^ and Immunoblot or Western blot tests.^3^, ^23^, ^24^, ^25^, ^40^ Some other tests were also used including; chemiluminescent magnetic microparticle immunoassay, enzyme‐linked fluorescence assay,^14^ HIV RT1 and RT2‐enzyme immunoassay,^24^ HIV viral load,^32^ and CD4 lymphocyte counts.^15^

### 4.6 HBV and HCV

In total, 18 studies‐ including two cross‐sectional studies assessed HCV infection,^22^, ^39^ five (one cohort study, and four cross‐sectional) studies investigated HBV infection^18^, ^20^, ^32^, ^33^, ^42^ and 10 articles evaluated both HBV and HCV infections^15^, ^17^, ^24^, ^25^, ^28^, ^35^, ^40^ used laboratory testing among prisoner participants.

According to CDC protocols, the gold standard for HBV infection testing is composed of HBsAg and anti‐HBc Ab IgM and IgG classes.^67^ Similarly, the main diagnostic test used for HBV diagnosis among included studies in this review is HBsAg, which was used in all HBV assessments through two methods; immunoassay in 13 studies, and rapid Ag test in two studies. Additionally, some studies also measured other serologic markers including anti‐HBc Ab (IgM and IgG), anti‐HBs Ab, HBeAg, anti‐HBe Ab, HBV‐DNA viral load to evaluate the infectivity, and severity of hepatitis B infection.^14^, ^17^, ^24^, ^25^, ^28^, ^40^, ^41^

In addition, based on CDC recommendations, the most sensitive and specific method for HCV infection testing includes the Anti‐HCV Ab test with HCV RNA nucleic acid test confirmation.^66^ In our study, the main laboratory diagnostic test for HCV was HCV immunoglobulin G (IgG) antibodies immunoassay (HCV IgG Ab) which was utilized in all HCV prevalence assessment included studies except for one study that had used chemiluminescent microparticle immunoassay^23^ and one other study that had utilized immunoblot kits.^25^

### 4.7 Syphilis

In our systematic review, 10 studies utilized laboratory tests to investigate possible Treponema pallidum infection among prisoners.^14^, ^15^, ^16^, ^17^, ^18^, ^24^, ^25^, ^32^, ^33^, ^40^ Rapid Plasma Reagin test was used in four studies,^14^, ^15^, ^32^, ^33^ six articles^14^, ^17^, ^18^, ^24^, ^33^, ^40^ used IgG, IgM, and IgA antibodies against Treponema pallidum, Treponema pallidum Micro‐hemagglutination assay^14^, ^15^ was used in two research studies and finally, Venereal Disease Research Laboratory^17^, ^40^ was used in two articles to detect syphilis infection.

### 4.8 Other STDs

Finally, four studies assessed the prevalence of other STDs including; Neisseria gonorrhea, Chlamydia trachomatis, and HSV‐2 by Anyplex CT/NG Seegene technique,^21^ GC/CT (urine sample, nucleic acid amplification test [NAAT]),^32^, ^33^ and HSV‐2 IgG (ELISA),^22^ respectively.

CDC recommends NAAT for routine use to screen and diagnose Chlamydia trachomatis and Neisseria gonorrhoeae among suspicious patients,^68^ and antibodies against HSV specific glycoproteins immunoassay for HSV testing and screening.^69^ To summarize, almost all the included studies met the diagnostic protocols recommended by the CDC.

### 4.9 STI prevalence

In total, 30 articles in our review reported the prevalence of different STIs among prisoners of various regions around the globe, there was significant heterogeneity in prevalence rates. In one similar systematic review that was conducted to assess the prevalence of HIV, HBV, and HCV infection rates among prisoners in Iran, the pooled prevalence rates were reported 2.77%, 2.89%, and 21.57%, respectively.^70^ Another systematic review carried out in Ethiopia among prisoners reported that the overall prevalence of HBV and HCV among prisoners was 22.3% and 4.3% respectively.^71^ Also, another study reviewed age differences in regard to the global prevalence of HBV, HCV, and HIV among incarcerated people and reported a range of 0.4%−25.2%, 0%−70.6%, and 0%−15.8%, respectively. They also reported that the rates of HCV infection were lower in younger inmates compared to older prisoners.^72^

Some studies included in our review described the gender differences regarding STD infection prevalence among prisoners; one study reported female rates of STD infections as follows; HIV 0.8%, HCV 2.6%, HBV 3.3%, and syphilis 3.3%, while male rates of STD infection were: HIV 0.7%, HCV 3.3%, HBV 2.9%, and syphilis 1.8%.^17^ Also, another study in our review reported that the prevalence of HCV was 31% and15.4% in males and females, respectively.^39^

One similar systematic review conducted in India among incarcerated participants reported that the prevalence of HBV and HCV in prisoners was 8% and 7% respectively. Regarding possible gender gaps, the prevalence rate of HBV and HCV among male prisoners was 4.48% and 6.35%, respectively, while the prevalence among female prisoners was 1.53% and 2.10%, respectively.^73^

One of the studies included in our review was conducted in Italy to investigate the coinfection rates of HBV and HCV among prisoners living with HIV‐1. The findings indicated a prevalence rate of 81.2% for HBV and HCV separately, whereas the prevalence of HBV/HCV coinfection was 69.6%.^41^ In Italy, one study carried out among 973 inmates, reported seroprevalences of HIV, HCV, anti‐HBc, HBsAg at 7.5%, 38.0%, 52.7%, and 6.7%, respectively. They also, found a strong association between HIV and HCV infection with intravenous drug use.^61^

A similar systematic review conducted to evaluate the prevalence of HBV and HCV coinfections among incarcerated people living with HIV reported a pooled prevalence rate of 12% for HBV‐HIV coinfection and 62% for HCV‐HIV coinfection. In addition, they emphasized that among HIV‐positive inmates with a history of drug injection, the prevalence rate of HBV and HCV increased to 15% and 78% respectively.^74^ A similar study in Nigeria among 300 incarcerates, reported 18.0%, 23.0% and 12.3% prevalence rates of HIV, HBV, and HCV, respectively, they also showed co‐infections rates of 2.7% and 0.7% for HIV/HBV and HBV/HCV, respectively. In the same study, they noted that younger inmates were at higher risk for HIV and HBV infection, while older prisoners had the highest HCV infection rates.^63^

One systematic review conducted among European countries, stated that in general, the highest HBV prevalence was among prisoners ranging from 0.3% to 25.2%, followed by IV drug users ranging from 0.5% to 6.1%, and similarly the highest prevalence HCV also was among prisoners ranging from 4.3% to 86.3%, and IV drug users ranging from 13.8% to 84.3%.^61^

One large study in Tehran, Iran among 6900 male inmates reported 85 HIV‐positive patients (1.23%), and indicated that age, imprisonment duration, history of injection drug use, history of sharing needles, and tattooing as the independent risk factors, associated with HIV infection.^75^ Another included study reported HIV as the most prevalent STD (0.68%), followed by Tuberculosis (0.66%), syphilis (0.2%), HCV (0.2%), and HBV (0.04%), and HIV‐syphilis coinfection.^24^ One similar study included in our review, conducted among confirmed tuberculosis prisoners reported a coinfection rate of 4.7% for HCV. Also, 19 TB cases were people living with HIV, 1.4% had chronic hepatitis B infection, lifetime syphilis infection was 10%, and active syphilis was 5%.^40^

## 5 CONCLUSION

Based on the findings of our review, the prevalence of STIs in prisoners including HIV, HBV, HCV, Syphilis, Chlamydia, Gonorrhea, and HSV‐2, was relatively higher than the general population. We also conclude that age, long prison sentences, low educational levels, poor knowledge of STIs, unsafe sexual activities, low condom use, IV drug abuse, needle sharing, tattooing, poor accessibility to preventive measures, single marital status as possible risk factors for developing STIs in prisons. Thus, to control the STIs prevalence in prisons, cost‐effective measures are necessary to be taken for limiting the risk factors, intensifying harm reduction programs, and enforcing global STI prevention guidelines in prisons.

## AUTHOR CONTRIBUTIONS

*Conceptualization and supervision*: Esmaeil Mehraeen, SeyedAhmad SeyedAlinaghi. *Data curation and investigation*: Zahra Pashaei and Ensiyeh Rahimi. *Methodology and formal analysis*: Solmaz Saeidi, Pegah Mirzapour. Writing – original draft preparation: Tayebeh Noori, Afsaneh Ghasemzadeh, ‎ Arian Afzalian, Mohsen Dashti, Pedram Habibi, Behnam Farhoudi, Narjes Aghaie, and Ahmadreza Shamsabadi. *Validation*: SeyedAhmad SeyedAlinaghi and Omid Dadras. Writing – review and editing: Esmaeil Mehraeen, Omid Dadras, and SeyedAhmad SeyedAlinaghi. All authors have read and approved the final version of the manuscript. Esmaeil Mehraeen had full access to all of the data in this study and takes complete responsibility for the integrity of the data and the accuracy of the data analysis.

## CONFLICT OF INTEREST

The authors declare no conflict of interest.

## TRANSPARENCY STATEMENT

The lead author Esmaeil Mehraeen affirms that this manuscript is an honest, accurate, and transparent account of the study being reported; that no important aspects of the study have been omitted; and that any discrepancies from the study as planned (and, if relevant, registered) have been explained.

## Data Availability

The authors stated that all information provided in this article could be share.
